RETRACTED

# Circular RNA ZNF609 drives tumor progression by regulating the miR-138-5p/SIRT7 axis in melanoma

**DOI:** 10.18632/aging.203394

**Published:** 2021-08-09

**Authors:** Quan Liu, Wei Cui, Chao Yang, Li-Ping Du

**Affiliations:** 1 Department of Plastic Surgery, Sichuan Academy of Medical Sciences and Sichuan Provincial People’s Hospital, Chengdu 610072, Sichuan, China; 2 Department of Traditional Chinese Medicine Surgery, Sichuan Academy of Medical Sciences and Sichuan Provincial People’s Hospital, Chengdu 610072, Sichuan, China

**Keywords:** melanoma, progression, DNA damage, circZNF609, miR-138-5p, SIRT7

## Abstract

Melanoma serves as a prevailing and lethal skin malignancy with high mortality and a growing number of patients globally. Circular RNAs (circRNAs), as a type of emerging cellular regulator, are involved in the modulation of melanoma. Nevertheless, the function of circZNF609 in melanoma development remains obscure. In this study, we were interested in the effect and the underlying mechanism of circZNF609 on DNA damage during melanoma progression. The circZNF609 depletion significantly suppressed melanoma cell invasion, migration, and proliferation, and stimulated apoptosis. Meanwhile, comet assays showed that the tail length and γH2AX levels were elevated by circZNF609 depletion. Mechanically, circZNF609 sponged miR-138-5p and miR-138-5p targeted SIRT7 in the melanoma cells. The SIRT7 overexpression and miR-138-5p inhibitor could reverse circZNF609 depletion-mediated DNA damage and malignant progression in melanoma cells. Functionally, CircZNF609 promoted cell growth of melanoma in the nude mice. Consequently, we conclude that circZNF609 suppresses DNA damage and potentially enhances melanoma progression at the experimental condition by modulating the miR-138-5p/SIRT7 axis. Our finding provides new insights into the mechanism by which circZNF609 modulates the development of melanoma. CircZNF609 and miR-138-5p may be utilized as therapeutic targets for melanoma.

## INTRODUCTION

Melanoma is a prevailing malignant skin cancer with high metastasis incidence and aggressive mortality, and the melanoma occurrence rate continues to increase globally [1–3]. In recent years, therapeutic strategies have advanced, but the prognosis of melanoma patients remains poor due to radiotherapy or chemotherapy resistance and metastasis [4]. In spite of advancement in diagnosis, such as the application of parallel reaction monitoring (PRM) and mass spectrometry [5], and the therapeutic strategy development, such as BRAF, CTLA4 and PD1 inhibitors [6, 7], the molecular mechanism of melanoma progression is still mostly unknown, which is urgently required to be further investigated [8, 9]. Some essential signaling pathways, including ERK signaling, NF-κB signaling, STING signaling, and WNT signaling, have been identified to present critical functions in melanoma development, and serve as important biomarkers for the diagnosis, prognosis, and treatment of melanoma [10–13]. According to the varied clinical features, melanoma can be divided as various types, such as follicular melanoma, mucosal melanoma, pigmented epithelioid melanocytoma, verrucous malignant melanoma, primary dermal melanoma, polypoid melanoma, and esemplastic melanoma [14]. Furthermore, DNA damage is a well-recognized cellular process and the therapeutic target for tumors and plays an essential function in melanoma development [15], but the molecular mechanisms of DNA damage in melanoma are elusive.

RETRACTED

Circular RNA (circRNA) is a kind of endogenous non-coding RNA with a covalent closed-loop structure [16], maintaining strong stability due to the exonucleolytic degradation resistance [5, 17]. With the advancement and development of RNA sequencing and RNA detection technology, circRNAs have been well-recognized to participate in various pathological and physiological processes, such as immune escape, cancer development, and tumorigenesis [18–20]. Meanwhile, several circRNAs have been found in the modulation of melanoma progression [21]. Moreover, circular RNA ZNF609 (circZNF609) is generated from the gene of ZNF609, which belongs to zinc finger family and is involved in the modulation of gene expression at DNA, RNA and protein levels [22]. CircZNF609 has been reported to play critical function in central nervous system. Recent studies revealed that circZNF609 is overexpressed not only in neurons, but also in various cancers, such as liver cancer, lung cancer, and prostate cancer [23–25]. Although the previous studies have shown that circZNF609 may serve as a crucial contributor to cancer development, the function of circZNF609 in melanoma development is still unreported. Accordingly, we were interested in the function of circZNF609 in the regulation of melanoma progression.

MicroRNAs (miRNAs) are stable single-stranded and small non-coding RNAs, demonstrating crucial functions in modulating cancer pathogenesis by targeting various genes at the post-transcriptional level [26, 27]. In the recent decade, it has been identified that miRNAs are involved in melanoma development and progression, regulating drug resistance of melanoma [28–31]. Meanwhile, miR-138-5p induces a tumor-suppressive effect on multiple cancers, including lung cancer, gastric cancer, and colorectal cancer [32–34]. Moreover, sirtuin 7 (SIRT7), as a deacetyltransferase, participates in the DNA damage process during tumorigenesis. However, the relationship of circZNF609 with SIRT7 and miR-138-5p remains unclear.

RETRACTED

Here, we aimed to explore the effect of circZNF609 on melanoma development *in vitro* and *in vivo*. We investigated the function of circZNF609 in DNA damage and melanoma phenotypes by MTT assays, Transwell assays, Wound healing assays, comet assays, flow cytometry analysis in A375 and SK-MEL-28 cells, and by tumorigenicity analysis in nude mice. The molecular mechanism was explored by bioinformatics analysis, qPCR, Western blot analysis, and luciferase reporter gene assays. We identified an unreported function of circZNF609 in repressing DNA damage and promoting melanoma cell proliferation by regulating miR-138-5p/SIRT7 axis.

## RESULTS

### CircZNF609 contributes to proliferation and attenuates apoptosis of melanoma cells

To assess the influence of circZNF609 on the cell proliferation of melanoma cells, the MTT assays and colony formation assays were performed in the A375 and SK-MEL-28 cells. The depletion of circZNF609 was able to reduce the viability of A375 and SK-MEL-28 cells (Figure 1A and 1B). Similarly, the colony formation of A375 and SK-MEL-28 cells was decreased by circZNF609 knockdown (Figure 1C and 1D). Meanwhile, the circZNF609 depletion significantly induced apoptosis of A375 and SK-MEL-28 cells (Figure 1E and 1F). Together these suggest that circZNF609 promotes proliferation and attenuates apoptosis of melanoma cells.

**Figure 1:** **CircZNF609 promotes proliferation and attenuates apoptosis of melanoma cells.** (**A**–**F**) The A375 and SK-MEL-28 cells were treated with the circZNF609 shRNA or control shRNA. (**A** and **B**) The cell viability was tested by the MTT assays in the cells. (**C** and **D**) The cell proliferation was measured by colony formation assays in the cells. (**E** and **F**) The cell apoptosis was analyzed by flow cytometry analysis in the cells. Data are presented as mean ± SD. Statistic significant differences were indicated: ^*^P < 0.05, ^**^P < 0.01, ^***^P < 0.001.

### CircZNF609 enhances invasion and migration of melanoma cells

Then, we further evaluated the role of circZNF609 in the migration/invasion of the melanoma cells. Transwell assay showed that the depletion of circZNF609 remarkably attenuated the migration and invasion of A375 and SK-MEL-28 cells (Figure 2A and 2B). In addition, wound healing assays revealed that the circZNF609 knockdown significantly enhanced wound proportion in the A375 and SK-MEL-28 cells (Figure 2C and 2D), suggesting that circZNF609 enhances invasion and migration of melanoma cells.

**Figure 2:** **CircZNF609 enhances invasion and migration of melanoma cells.** (**A**–**D**) The A375 and SK-MEL-28 cells were treated with the circZNF609 shRNA or control shRNA. (**A** and **B**) The cell migration and invasion were tested by transwell assays in the cells. (**C** and **D**) The migration and invasion were analyzed by wound healing assays in the cells. The wound healing proportion was shown. Data are presented as mean ± SD. Statistic significant differences were indicated: ^*^P < 0.05, ^**^P < 0.01.

RETRACTED

### CircZNF609 inhibits DNA damage in melanoma cells

Next, we determined the impact of circZNF609 on the DNA damage in the A375 and SK-MEL-28 cells. The comet assays showed that the tail length was increased by circZNF609 depletion in the A375 and SK-MEL-28 cells (Figure 3A and 3B). Meanwhile, γH2AX expression was up-regulated by circZNF609 shRNA in the A375 and SK-MEL-28 cells (Figure 3C and 3D), indicating that circZNF609 inhibits DNA damage in melanoma cells.

**Figure 3:** **CircZNF609 inhibits DNA damage in melanoma cells.** (**A**–**D**) The A375 and SK-MEL-28 cells were treated with the circZNF609 shRNA or control shRNA. (**A** and **B**) The DNA damage was analyzed by comet assays in the cells. (**C** and **D**) The protein expression of H2AX, γH2AX and β-actin was determined by Western blot analysis in the cells. The results of Western blot analysis were quantified by ImageJ software. Data are presented as mean ± SD. Statistic significant differences were indicated: ^*^P < 0.05, ^**^P < 0.01.

### CircZNF609 represses DNA damage by sponging miR-138-5p in melanoma cells

Next, we tried to explore the mechanism of circZNF609-mediated melanoma. We found the interaction between circZNF609 and miR-138-5p in a bioinformatic analysis by using ENCORI (starbase.sysu.edu.cn) (Figure 4A). Then, we treated the A375 and SK-MEL-28 cells with control mimic or miR-138-5p mimic, and the efficiency was confirmed in the cells (Figure 4B). The miR-138-5p mimic significantly inhibited the luciferase activities of circZNF609but failed to affect the circZNF609 with the miR-138-5p-binding site mutant in the cells (Figure 4C and 4D). Meanwhile, the depletion of circZNF609 was able to reduce the expression of miR-138-5p in the A375 and SK-MEL-28 cells (Figure 4E and 4F). Moreover, the comet assays revealed that the tail length was enhanced by circZNF609 depletion in the A375 and SK-MEL-28 cells, while the miR-138-5p inhibitor blocked the phenotype (Figure 4G and 4H). Besides, γH2AX expression was elevated by circZNF609 shRNA in the A375 and SK-MEL-28 cells, in which the miR-138-5p inhibitor reversed this effect (Figure 4I and 4J).

**Figure 4:** **CircZNF609 inhibits DNA damage by sponging miR-138-5p in melanoma cells.** (**A**) The interaction of circZNF609 and miR-138-5p was analyzed by bioinformatic analysis based on ENCORI (starbase.sysu.edu.cn). (**B**–**D**) The A375 and SK-MEL-28 cells treated with control mimic or miR-138-5p mimics. The expression levels of miR-138-5p were tested by qPCR in the cells. (**C** and **D**) Luciferase activities of circZNF609 (circZNF609 WT) and circZNF609 with the miR-138-5p-binding site mutant (circZNF609 MUT) were examined by luciferase reporter gene assays in the cells. (**E** and **F**) The A375 and SK-MEL-28 cells were treated with the circZNF609 shRNA or control shRNA. The expression of miR-138-5p was analyzed by qPCR assays in the cells. (**G**–**J**) The A375 and SK-MEL-28 cells were treated with the control shRNA or circZNF609 shRNA, or co-treated with circZNF609 shRNA and miR-138-5p inhibitor. (**G** and **H**) The DNA damage was analyzed by comet assays in the cells. (**I** and **J**) The protein expression of H2AX, γH2AX and β-actin was determined by Western blot analysis in the cells. The results of Western blot analysis were quantified by ImageJ software. Data are presented as mean ± SD. Statistic significant differences were indicated: ^*^P < 0.05, ^**^P < 0.01.

RETRACTED

### MiR-138-5p induces DNA damage by targeting SIRT7 in melanoma cells

Next, the miR-138-5p -targeted site in SIRT7 3′UTR was found by a bioinformatic analysis using Targetscan (http://www.targetscan.org/vert_72/) (Figure 5A). The miR-138-5p mimic repressed luciferase activities of wild type SIRT7 but failed to affect the SIRT7 with the miR-138-5p-binding site mutant in the A375 and SK-MEL-28 cells (Figure 5B). The mRNA expression of SIRT7 was decreased by miR-138-5p mimic in the cells (Figure 5C). Similarly, the protein expression of SIRT7 was inhibited by miR-138-5p mimic in the cells (Figure 5D). In addition, miR-138-5p inhibitor could rescue the circZNF609 depletion-inhibited SIRT7 expression (Figure 5E). Furthermore, the comet assays showed that the tail length was increased by miR-138-5p mimic in the A375 and SK-MEL-28 cells, while the SIRT7 overexpression inhibited the phenotype (Figure 5F and 5G). Similarly, the expression levels of γH2AX were enhanced by miR-138-5p mimic in the cells, in which SIRT7 overexpression could reverse this effect (Figure 5H and 5I), indicating that miR-138-5p induces DNA damage by targeting SIRT7 in melanoma cells.

**Figure 5:** **MiR-138-5p induces DNA damage by targeting SIRT7 in melanoma cells.** (**A**) The binding of miR-138-5p and SIRT7 3’UTR was identified by bioinformatic analysis based on Targetscan (http://www.targetscan.org/vert_72/). (**B**–**D**) The A375 and SK-MEL-28 cells were treated with control mimic or miR-138-5p mimic. (**B**) The luciferase activities of wild type SIRT7 (SIRT7 WT) and SIRT7 with the miR-138-5p-binding site mutant (SIRT7 MUT) were examined by luciferase reporter gene assays in the cells. (**C**) The mRNA expression of SIRT7 was analyzed by qPCR assays in the cells. (**D**) The protein expression of SIRT7 was determined by Western blot analysis in the cells. (**E**) The A375 and SK-MEL-28 cells were treated with control shRNA or circZNF609 shRNA, or co-treated with circZNF609 shRNA and miR-138-5p inhibitor. The protein expression of SIRT7 was tested by Western blot analysis in the cells. (**F**–**I**) The A375 and SK-MEL-28 cells were treated with the control mimic or miR-138-5p mimic, or co-treated with miR-138-5p mimic and pcDNA3.1-SIRT7. (**F** and **G**) The DNA damage was analyzed by comet assays in the cells. (**H** and **I**) The protein expression of H2AX, γH2AX and β-actin was determined by Western blot analysis in the cells. The results of Western blot analysis were quantified by ImageJ software. Data are presented as mean ± SD. Statistic significant differences were indicated: ^*^P < 0.05, ^**^P < 0.01.

RETRACTED

### CircZNF609 contributes to melanoma cell survival by miR-138-5 /SIRT7 axis

Next, we investigated the effect of the circZNF609/ miR-138-5p/ SIRT7 axis in melanoma development *in vitro*. MTT assays showed that the depletion of circZNF609 significantly reduced the viability of A375 and SK-MEL-28 cells, in which the miR-138-5p inhibitor or SIRT7 overexpression could rescue the phenotype (Figure 6A and 6B). Moreover, the cell apoptosis of A375 and SK-MEL-28 cells was induced by circZNF609 knockdown, while the miR-138-5p inhibitor or SIRT7 overexpression was able to reverse this effect (Figure 6C and 6D).

**Figure 6:** **CircZNF609 contributes to melanoma cell survival by miR-138-5p/SIRT7 axis.** (**A**–**D**) The A375 and SK-MEL-28 cells were treated with control shRNA or circZNF609 shRNA, co-treated with circZNF609 shRNA and miR-138-5p inhibitor or pcDNA3.1-SIRT7. (**A** and **B**) The cell viability was measured by MTT assays in the cells. (**C** and **D**) The cell apoptosis was analyzed by flow cytometry analysis in the cells. Data are presented as mean ± SD. Statistic significant differences were indicated: ^*^P < 0.05, ^**^P < 0.01.

### CircZNF609 promotes tumor growth of melanoma cells *in vivo*

We then examined the effect of circZNF609 on the melanoma *in vivo* by the tumorigenicity analysis of nude mice. Significantly, the depletion of circZNF609 remarkably reduced the tumor size, tumor volume, and tumor weight of the A375 cells in the mice (Figure 7A–7C). In addition, the expression of miR-138-5p was enhanced but the expression of SIRT7 was reduced by the circZNF609 knockdown in the tumor tissues of the mice (Figure 7D and 7E). Together these indicate that circZNF609 promotes tumor growth of melanoma cells *in vivo*.

RETRACTED

**Figure 7:** **CircZNF609 promotes tumor growth of melanoma cells *in vivo*.** (**A**–**D**) The impact of circZNF609 on tumor growth of melanoma cells *in vivo* was analyzed by nude mice tumorigenicity assay (*n* = 5). The A375 cells were treated with control shRNA or circZNF609 shRNA. (**A**) Representative images of dissected tumors from nude mice were shown. (**B**) The average tumor volume was calculated and presented. (**C**) The average tumor weight was calculated and presented. (**D**) The expression of miR-138-5p was measured by qPCR in the tumor tissues of the mice. (**E**) The expression of SIRT7was tested by Western blot analysis in the tumor tissues of the mice. Data are presented as mean ± SD. Statistic significant differences were indicated: ^*^P < 0.05, ^**^P < 0.01.

## DISCUSSION

Melanoma serves as a prevalent skin cancer, in which the patients hold poor prognosis and survival rates [35]. Although the advancements in surgery, chemotherapy, radiotherapy, metastasis, and drug resistance are still the leading reason for melanoma-induced mortality, and understanding the molecular mechanism of melanoma development is urgently required [36]. CircRNAs have presented fundamental functions during cancer progression. In this study, we uncovered that circZNF609 inhibited DNA damage and enhanced melanoma development by miR-138-5p/SIRT7 axis.

As an emerging biological modulator, many circRNAs have been reported to regulate melanoma progression. It has been reported that circITCH inhibits glucose uptake to repress cell proliferation by down-regulating GLUT1 expression in melanoma [37]. Circ0020710 enhances immune evasion and tumor development of melanoma by the modulation of miR-370-3p/CXCL12 signaling [38]. Circ0017247 contributes to invasion and migration of melanoma cells by regulating miR-145 [39]. Circular RNA circ_0079593 contributes to the progression of melanoma by targeting miR-573/ABHD2 signaling [40]. Circ0001591 promotes metastasis and proliferation of melanoma cells by targeting miR-431-5p-mediated ROCK1/PI3K/AKT signaling [41]. These reports indicate that circRNAs play crucial roles in the modulation of melanoma. Our results demonstrated that circZNF609 promoted cell proliferation/migration/invasion, and inhibited apoptosis of melanoma cells. CircZNF609 was able to repress DNA damage in melanoma cells. CircZNF609 enhanced melanoma cell growth *in vivo.* These data elucidate a new function of the circZNF609 for regulating DNA damage and progression during melanoma pathogenesis, presenting informative evidence of the role of circRNAs in melanoma development. Meanwhile, due to that DNA damage plays critical roles in the pathogenesis of aging-related diseases, the function in the regulation of aging-related diseases and senescence-related markers should be explored in future studies. Given that the crucial role of circZNF609 in promoting the malignant progression of melanoma, targeting circZNF609 may serve as a promising therapeutic strategy for the treatment of melanoma. Meanwhile, the expression of circZNF609 in clinical melanoma samples and the serum samples of melanoma patients and the correlation of circZNF609 with the clinical characteristics of melanoma should be identified by more investigations. Based on the critical function of circZNF609 and the clinical correlation with melanoma, the diagnostic and prognostic significance of circZNF609 will be identified and circZNF609 may serve as a potential biomarker for melanoma. Moreover, the investigations of the interaction between circular RNAs, including circZNF609 and other types of circular RNAs, are limited and should be explored in the future.

RETRACTED

MiRNAs are the fundamental factors for post-transcriptional regulation of various targeted genes in melanoma development [28]. It has been reported that miR-489-3p/SIX1 axis controls the cell proliferation and glycolytic potential during melanoma progression [42]. MiR-33a-5p suppresses the metastasis and growth by the modulation of SNAI2 expression in melanoma cells [43]. MiR-410-3p activated by ER stress is responsible for the BRAF inhibitor resistance in melanoma [30]. These studies indicate that miRNAs are widely involved in the modulation of melanoma. In addition, it has been found that cancer-delivered exosomal miR-138-5p regulates polarization of tumor-associated macrophage by inhibiting KDM6B [44]. MiR-138-5p regulates the ERCC4 and ERCC1 expression in gastric cancer cells, contributing to the cisplatin sensitivity [33]. MiR-138-5p is involved in Long non-coding RNA MCM3AP-AS1/FOXK1 promoted migration and growth of pancreatic cancer [45]. These investigations indicate that miR-138-5p serves as potential tumor suppression by targeting various genes. Moreover, previous studies have identified that SIRT7 regulates deacetylation of ATM and participates in DNA damage repair in cancer cells [46]. SIRT7 is able to modulate deacetylation of H3K18 in regulating DNA damage [47]. Our mechanism exploration showed that circZNF609 inhibited DNA damage by sponging miR-138-5p and miR-138-5p enhanced DNA damage by targeting SIRT7 in melanoma cells. The SIRT7 overexpression and miR-138-5p inhibitor could reverse circZNF609 depletion-mediated DNA damage and malignant progression in melanoma cells. These data reveal an unreported correlation of circZNF609 with miR-138-5p and SIRT7 in the modulation of melanoma, demonstrating a new molecular mechanism involving circZNF609/miR-138-5p/SIRT7 axis in melanoma. In this study, we identified that SIRT7 was involved in the circZNF609/miR-138-5p signaling-mediated melanoma. These results are consistent with the previous reports about SIRT7 regulates DNA damage and contributes to melanoma development. The inhibitors of SIRT7 may become the potential candidates for the treatment of melanoma and should be developed in future basic and clinical investigations. Meanwhile, in the present study, we identified that miR-138-5p served as a potential tumor suppression in melanoma. As the miRNA-based anti-tumor strategies have been developed for many years, the delivery and target system for miR-138-5p in the treatment of melanoma need to be explored in future. Due to that miRNAs have presented the diagnostic and prognostic values in cancers, the clinical expression and significance of miR-138-5p should be identified by further studies.

RETRACTED

Consequently, we concluded that circZNF609 suppressed DNA damage and potentially contributed to melanoma development in the experimental condition by modulating the miR-138-5p/SIRT7 axis. CircZNF609 and miR-138-5p may be utilized as the therapeutic targets for melanoma.

## METHODS

### Cell culture and treatment

We evaluated the effect of circZNF609 on melanoma *in vitro* using SK-MEL-28 and A375 cells. The SK-MEL-28 and A375 cells were incubated at 37°C and 5% CO_2_ in FBS (10%, Hyclone, USA) and streptomycin (0.1 mg/mL, Hyclone, USA)/penicillin (100 units/mL, Hyclone, USA)-supplemented RPMI 1640 medium. The control shRNA, circZNF609 shRNA, pcDNA3.1-SIRT7, miR-138-5p mimic/inhibitor were synthesized (GenePharma, China). Liposome 2000 (Invitrogen, USA) was utilized for the transfection.

### RNA extraction and RT-qPCR

We measured the expression of circZNF609, miR-138-5p, and SIRT7 by RT-qPCR analysis in the SK-MEL-28 and A375 cells and tumor tissues. After 48 hours of the indicated treatment in SK-MEL-28 and A375 cells, the TRIZOL (Invitrogen, USA) was utilized to extract total RNAs from the cells and RNAs were subjected to first-strand cDNA synthesis (TaKaRa, China). The qPCR was carried out using SYBR-Green (Takara, China). The experiments were performed at least 3 times independently. CAPDH and U6 were used as internal control for normalization of mRNA and the noncoding RNAs. The relative change in RNA levels were calculated by 2^−ΔΔCt^ method. The primers information: circZNF609 forward: 5′-CATGCTGATTACGCTTTGACTC-3′, reverse: 5′-GTTTCGTTCATCTGCTACTT-3′; miR-138-5p forward: 5′-AGCTGGTGTTGTGAATCAGGCCG-3′, reverse: 5′-TGGTGTCGTGGAGTCG-3′; SIRT7 forward: 5′-GAGAGCGAGGACCTGGTGAC-3′, reverse: 5′-GATAGAGGCTGCCGTGCTGA-3′; GAPDH forward: 5′-AAGAAGGTGGTGAAGCAGGC-3′, reverse: 5′-TCCACCACCCAGTTGCTGTA-3′; U6 forward: 5′-GCTTCGGCAGCACATATACTAA-3′, reverse: 5′-AACGCTTCACGAATTTGCGT-3′.

RETRACTED

### MTT assay

We examined the activity of circZNF609 on A375 and SK-MEL-28 cell viability using MTT assays. The A375 and SK-MEL-28 cells were conducted with indicated treatment, and cells were seeded in 96-well plates at a density of 4 × 103 cells per well to growth for 48 hours and treated with MTT (Solarbio, China) at the indicated time, followed by 4-hours incubation. The 100 μL dimethyl sulfoxide (DMSO, Sigma, USA) was used to terminate the reaction and the results were read using microplate reader (490 nm, Thermo, USA).

### Colony formation

We detected the function of circZNF609 in A375 and SK-MEL-28 cell proliferation using colony formation analysis. After 48 hours of the indicated treatment in SK-MEL-28 and A375 cells, the A375 and SK-MEL-28 cells (1 × 10^3^) were plated in 6-well plates, and maintained in normal culture condition to allow formation of mono colonies. After incubation for 12 days, the colonies were fixed and stained by 0.5% crystal violet in methanol for 30 minutes. The colonies were captured under a microscope (Olympus, Japan) and counted.

### Transwell assays

We determined the role of circZNF609 in invasion and migration using transwell assays in A375 and SK-MEL-28 cells treated as the indication. To analyze cell invasion, the Matrigel (BD, USA)- coated chambers were plated with the cells (1 × 10^5^) and serum-free medium was added. The bottom chambers were fixed with complete medium. The cells were dyed using crystal violet and counted. The migration analysis used the similar procedure without Matrigel.

### Wound healing assay

We assessed the circZNF609-mediated A375 and SK-MEL-28 cell migration using wound healing assays. A375 and SK-MEL-28 cell cells were transfected with as the indication for 48 hours and cells (3 × 10^5^/well) were plated in 24-well plates to form a monoplayer. A sterilized 200 ul pipette were used to gently scratch a line on the monoplayer. Then the cells were washed with PBS to wash out the detached cells, and replaced with fresh FBS-free medium for continuing incubation. The images of scratch were captured at 0 h, 6 h and 12 h after scratching with a microscope (Olympus), and measured.

### Analysis of cell apoptosis

We evaluated the circZNF609-induced A375 and SK-MEL-28 cell apoptosis using Annexin V-FITC Apoptosis Detection Kit (keygen, China). A375 and SK-MEL-28 cell cells were planted in 6-well plate at a density of 2 × 105/well, and conducted with indicated treatment for 48 hours. Next, the cells were digested with EDTA-free trypsin to single-cell and collected, followed by re-suspension in binding buffer and incubation with PI and Annexin-FITC at room temperature for 15 minutes in dark. Then the suspension was detected in a Flow cytometry (BD bioscience, USA) to collect fluorescence signals.

RETRACTED

### Comet assays

The DNA damage was analyzed by comet assays. Shortly, A375 and SK-MEL-28 cells treated as the indication for 48 hours were resuspended and added with to low-melting agarose (0.7%, 250 μL at 37°C, ice condition, 10 minutes), followed by alkaline lysis buffer (overnight, 4°C). After that, the cells were cultured in alkaline electrophoresis buffer (30 minutes) followed by the running (electrophoresis buffer, 23 V, 300 mA, 30 minutes) based on the Comet Assay tank (Thistle Scientific, UK). For the DNA staining, the cells were dyed with PI (50 μM, 10 minutes). The DNA damage was observed using fluorescence microscope and the tail length was calculated by applying CometScore software.

### Dual Luciferase reporter assays

The potential binding sites between miR-27a-3p with CircFNDC3B or 3′UTR of YAP were predicted by online website ENCORI. The wide type and mutated sequence of circZNF609 (circZNF609-WT and circZNF609-Mut) and 3′UTR of SIRT7 (SIRT7-WT and SIRT7-Mut) were inserted into psiCHECK2 plasmid (Promega, WI, USA). A375 and SK-MEL-28 cells were planted in 24-well plate at a density of 2 × 105/well, followed by co-transfection with indicated luciferase reporter plasmids and miR-138-5p mimics or the negative control (NC) for 48 hours. Then the cells were collected and lysed, and the luciferase activity was measured by the dual-luciferase reporter assay system (Promega, WI, USA) following the manufacture’s instruction. The results were normalized to Renilla luciferase activity.

### Western blot analysis

We measured the expression of yH2AX, H2AX, and SIRT7 using Western blot. The cell lysate in A375 and SK-MEL-28 cells treated as the indication for 48 hours and the tumor tissues was collected using RIPA buffer (CST, USA) and the protein concentration was determined by BCA Protein Quantification Kit (Abbkine, USA). The samples were subjected into SDS-PAGE, transferred to PVDF membranes (Millipore, USA), and blocked using skim milk (5%) for 2 hours at 25°C. The membrane was incubated with anti-H2AX antibodies (Abcam, USA), anti-γH2AX antibodies (Abcam, USA), anti-SIRT7 antibodies (Abcam, USA), and anti-β-actin antibodies (Abcam, USA) overnight at 4°C, and secondary antibodies (Abcam, USA) for 1 hour at 25°C, respectively. The results were observed by applying chemiluminescence detection kit (Beyyotime, China).

RETRACTED

### Tumorigenicity analysis

We analyzed the impact of circZNF609 on melanoma cell growth *in vivo* using the tumorigenicity analysis in Balb/c nude mice (4-weeks-old, male, *n* = 5). The mice were subcutaneously injected with control shRNA or circZNF609 shRNA treated A375 cells. The tumor length/width and mice weight were monitored every five days after injection of five days. The mice were euthanized after thirty days of injection. The method of (L × W^2^) × 0.5 was applied to calculate tumor volume. The experiments conformed to the authorization of Animal Ethics Committee of Sichuan Provincial People’s Hospital (Approval No. 2020-0319-17).

### Statistical analysis

The GraphPad prism 7 was applied for the statistical analysis and the results were reported by mean ± SD. Two of multiple groups differences were compared using Student’s *t*-test and one-way ANOVA, respectively, and *P* < 0.05 was statistically significant.
